# Relationship between Acute Mastitis and Constitution of Traditional Chinese Medicine in Chinese Breastfeeding Mothers

**DOI:** 10.1155/2021/2255511

**Published:** 2021-10-13

**Authors:** Yijia Bao, Jingyi Hu, Yuenong Qin

**Affiliations:** ^1^Integrated Chinese and Western Medicine Department of Breast Surgery, Longhua Hospital, Affiliated Hospital of Shanghai University of Traditional Chinese Medicine, Shanghai, China; ^2^Gaojing Town Community Health Center, Baoshan District, Shanghai, China

## Abstract

**Objective:**

The purpose of this study was to explore the relationship between acute mastitis and the constitution of traditional Chinese medicine (TCM) and the potential risk factors of acute mastitis in Chinese breastfeeding mothers.

**Method:**

A retrospective study on infant feeding practices was conducted in the Breast Surgery Department of Longhua Hospital Affiliated to Shanghai University of Traditional Chinese Medicine between February 2017 and March 2018. A total of 184 women with acute mastitis and 201 women without mastitis of childbearing age were included in this study. All participants filled a baseline questionnaire on demographic characteristics, previous deliveries, and mastitis history and other possible risk factors; data were collected by face-to-face interview. Logistic regression analysis was conducted to ascertain pertinent risk factors affecting the incidence of acute mastitis. The biased constitution of TCM of participants was identified through questionnaires surveyed with the TCM constitution table (ZYYXH/T157-2009). The relationship between acute mastitis and the constitution of TCM was assessed.

**Results:**

The protective factors included regular nipple cleansing and cesarean section. The risk factors were nipple infection, Primipara, improper diet, emotional stimuli, postpartum colostrum overdue for more than 72 h, breastfeeding more than 7 times each day, and late primiparity age. Forty-five percent of acute mastitis occurred within 8 weeks after postpartum, and the most common biased constitution of TCM at this period was Qi-Deficiency Constitution (QDC) and Qi-Stagnation Constitution (QSC). Another peak was 25–48 weeks after delivery, accounting for 18%, and the most common biased constitution of TCM was QSC and QDC. More participants were or were prone to be classified as Balanced Constitution (BC) in the control group than the case group (88.5% vs 29.6%), while QDC was the most common constitution of TCM in the case group. The logistic regression analysis further proved that BC was the protective factor of acute mastitis while QDC was a risk factor.

**Conclusions:**

The protective factors of acute mastitis were regular nipple cleansing and cesarean section. The risk factor was nipple infection. Among all the constitutions of TCM, BC was a protective factor, while QDC was a risk factor. For all breastfeeding mothers with various constitutions of TCM, regular nipple cleansing and breast vacuuming, a healthy lifestyle, and a positive mental state can keep mastitis away.

## 1. Introduction

Mastitis is an inflammation condition of the breast tissue [1]. It is clinically characterized by a tender, hot, and swollen wedge-shaped area of the breast in conjunction with influenza-like symptoms, such as fever and malaise [2]. In some cases, untreated or inadequately treated mastitis can develop into breast abscesses or septicemias [3]. The incidence of acute mastitis in breastfeeding mothers ranges from 3% to 40%, and about 17% to 33% of foreign mothers suffer from acute mastitis in breastfeeding [4–10]. Nipple trauma, especially if *Staphylococcus aureus* is colonized, has been known to induce mastitis [7]. Other risk factors, including maternity status, such as parity, primiparity age, and delivery mode [4, 12], lactation-related factors, such as first lactation time, daily lactation time, and milk yield [11–13], and mental condition [4] may also contribute to mastitis. The key components of management are symptom control, oral antibiotics, and encouraging continued milk flow from the affected breast. Close monitoring is required to ensure that the infection is resolved [7].

Unlike that in Western countries, there are few studies about lactation mastitis in Asian women. Therefore, few extensive researches and published literature focused on acute mastitis in Chinese women. Late marriage and late childbearing are more and more common in China, especially in first-tier cities [14]. Moreover, differences in postpartum care practices between East and West may also lead to a different prevalence of acute mastitis.

The theory of the constitution of traditional Chinese medicine (TCM) can be traced back to the Han Dynasty, and it was officially announced and well-defined in the 1970s [15]. In the past 40 years, this theory has been supplemented by applying modern technology or new algorithms. The research of the constitution of TCM can guide the individual treatment and prevention of diseases and also can judge the prognosis and susceptibility of diseases. Therefore, we applied questionnaires about the constitution of TCM to identify the susceptible constitution of TCM as well as the relationship between the incidence of acute mastitis and the constitution of TCM in Chinese breastfeeding mothers.

## 2. Subjects and Methods

### 2.1. Subjects

All participants signed informed consent. A retrospective study on infant feeding practices was conducted in the Breast Surgery Department of Longhua Hospital Affiliated to Shanghai University of Traditional Chinese Medicine between February 2017 and March 2018. A total of 184 women with acute mastitis and 201 women without mastitis of childbearing age were included in this study. They were all involved in the study of mastitis-related risk factors between February 2017 and January 2018. In addition, 162 women with acute mastitis and 104 women without mastitis of childbearing age were involved in the study of the relationship between the incidence of acute mastitis and the constitution of TCM between June 2017 and March 2018.

Inclusion criteria: women with acute mastitis were included in the following criteria: (i) postpartum breastfeeding women who met the diagnostic criteria, (ii) patients who were newly diagnosed with acute mastitis in Longhua Hospital, and (iii) patients who completed informed consent and related notification. The women without acute mastitis were included in the following criteria: (i) women who had been breastfeeding and had not been affected by diseases and (ii) women who were 18–45 years old. Exclusion criteria: women with acute mastitis were excluded in the following criteria: (i) pregnant women or postpartum women who did not breastfeed infants, (ii) women who had a history of breast cancer or diagnosed as inflammatory breast cancer, (iii) serious mental diseases, (iv) mentally challenged or mental retardation, and (v) serious heart, lung, and kidney diseases with limited life expectancy. The women without acute mastitis were excluded in the following criteria: (i) women who had a history of acute mastitis, (ii) women who have already bear children but did not breastfeed infants, (iii) serious mental disease, (iv) mentally challenged or mental retardation, and (v) serious heart, lung, and kidney diseases with limited life expectancy.

### 2.2. Case Definition

The definition of “acute mastitis” was adopted from the previous literature [13]. Mastitis was defined as the symptoms of a pink, tender, hot, swollen area of the breast, accompanied by one or more of the following: (i) an elevated temperature, (ii) one of the constitutional symptoms of fever (body aches, headaches, and chills), and (iii) diagnosis of mastitis by a medical practitioner. Symptoms must be present for a minimum duration of 24 h [13, 16]. Acute mastitis can be divided into two phases: stagnation stage and suppurative stage according to the Practical Traditional Chinese Medicine Surgery [17]. Symptoms in the stagnation period are swelling and pain of the breast, with or without mass, insufficient secretion of milk, or reddish skin. In the suppurative stage, symptoms are the breast obvious mass, the reddish skin, the pain of continuous jumping, fever and shivering, headache, and bone pain.

### 2.3. Questionnaires

The women completed a baseline questionnaire on demographic characteristics, previous deliveries, history of mastitis, and other possible risk factors. After participants filled out the whole questionnaires, the questionnaires were recovered on the spot. Risk factors in the questionnaire included general physical condition, breastfeeding condition, maternal condition, and mastitis symptoms. The biased constitution of TCM of participants was identified through questionnaires surveyed with the TCM constitution table (ZYYXH/T157-2009) published by the China Association of Chinese Medicine in 2009 ^[18]^. The single choice of “TCM Constitution Classification and Judgment Self-Test Table” in each question option scores from “no” to “often” as 1 to 5 points, respectively (Table 1). We calculated the original score and record the corresponding conversion score and constitution of TCM by

(1) $$\begin{array}{c} \text{Conversion Score}=\;\left[\frac{\left(\text{Original Score}-\text{Item Number}\right)}{\left(\text{Item Number}*4\right)}\right]*100. \end{array}$$

### 2.4. Definition of Risk Factor Exposure

The demographic characteristics and clinical characteristics were obtained from the baseline questionnaire. For breastfeeding mothers with mastitis, data on potential risk factors were based on the information recorded before their first episode of mastitis. For women who did not develop mastitis, data were taken from the questionnaire administered prior to the cessation of breastfeeding.

### 2.5. Statistical Analysis

Statistical analysis was made by software SPSS 21.0 (International Business Machines, corp., Armonk, NY, USA). Descriptive statistics were first applied to analyze the characteristics of participants. We assessed the distribution of demographic factors, career-related factors, fertility, and breastfeeding-related factors between women with acute mastitis and without acute mastitis, and the differences between the two groups were tested by using the *Chi-square* test and *t*-test. Logistic regression analysis and cluster analysis were conducted to extract potential risk factors affecting the incidence of mastitis and to identify the correlation between the constitution of biased TCM and the incidence of acute mastitis. Independent variables considered in the regression model were plausible risk factors from the literature. Both odd ratio (OR) and corresponding 95% confidence intervals (CIs) were used to assess the magnitude of the associations. Differences were considered statistically significant when *p* < 0.05.

## 3. Results

### 3.1. Baseline Demographic Characteristics and Clinical Characteristics

We established an acute mastitis cohort including 184 patients with acute mastitis and a control cohort including 201 healthy women with similar average ages and educational backgrounds (Table 2).

The age of the case group was 31.13 ± 3.62 years, and that of the control group was 32.09 ± 4.19 years. The baseline data of the two groups were balanced. The age at the first birth of the case group was 31 ± 4 years, and that of the control group was 28 ± 3 years. A total of 162 patients with acute mastitis and 102 healthy women were included in the study of the correlation between the constitution of biased TCM and the incidence of acute mastitis. All participants completed the “Self-Test Form for Classification and Judgment of TCM Constitution”. The age of the case group was 31.11 ± 3.63 years, and that of the control group was 30.49 ± 3.37 years. The baseline data of the two groups were balanced.

### 3.2. The Prevalence of Acute Mastitis in the Case Group

Of all 184 patients, 82 patients (44.6%) occurred in the left side of breasts, 84 patients (45.7%) occurred in the right side of breasts, and 18 patients (9.8%) occurred on both sides. The duration of mastitis was less than 3 days in 126 patients (68.5%), 4–7 days in 35 patients (19.0%), 8–14 days in 15 patients (8.2%), 15–21 days in 5 patients (2.7%), and more than 21 days in the remaining 3 patients (1.6%). 176 patients (95.7%) were at the stagnation stage, while only 8 of them (8.3%) were at the suppurative stage during the follow-up period.

When analyzing the onset time of acute mastitis, we found that acute mastitis usually occurred within 8 weeks after delivery, accounting for 45% of the total sample size, followed by 25–48 weeks after delivery, accounting for 18% (Figure 1).

### 3.3. The Risk Factors Affecting Incidence of Acute Mastitis

The results of Chi-square tests showed that parity, primiparity age, fetal status, postpartum colostrum, first lactation time after delivery, times of lactation each day, time of consecutive feeds with the same breast, and times of nipple cleansing each day in the case group were statistically significant in comparison with those in the control group (Table 3). According to the results of our preliminary experiment and related factors adopted from the previous literature, improper diet, emotional stimulation, and delivery mode were considered to be relevant to the occurrence of acute mastitis and were taken into account, although the contribution of delivery mode was quite controversial. Therefore, 11 possible related risk factors, including primiparity age, mode of delivery, postpartum colostrum, first lactation time after delivery, times of breastfeeding each day, time of consecutive feeds with the same breast, frequency of nipple cleansing, nipple infection, improper diet, and emotional stimulation, were extracted from the questionnaire as statistically related factors and the rest were observational factors.

After introducing 11 possible related risk factors, 9 risk factors, including primiparity age, mode of delivery, postpartum colostrum, times of breastfeeding each day, frequency of nipple cleansing, nipple infection, improper diet, stress, and parity, were screened by Forward Stepwise Regression. The OR value and its 95% CI of “nipple infection” were 7.128 and (3.804, 13.357), respectively, so it can be considered as a risk factor for the occurrence of acute mastitis. In addition, primiparity (OR: 5.053; 95%CI: 2.107, 12.118), improper diet (OR: 3.573; 95%CI: 1.967, 6.488), stress (OR: 1.930; 95%CI: 1.059, 3.519), postpartum colostrum (OR: 1.742; 95%CI: 1.283, 2.364), times of breastfeeding each day (OR: 1.475; 95%CI: 1.036, 2.100), and late primiparity age (OR: 1.135; 95%CI: 1.050, 1.226) were also risk factors for the occurrence of acute mastitis. Cesarean section (OR: 0.540; 95%CI: 0.322, 0.910) and frequency of nipple cleansing (OR: 0.484; 95%CI: 0.350, 0.671) can be considered as protective factors for the occurrence of acute mastitis. However, there were no significant correlations between the first breastfeeding time after delivery, time of consecutive feeds with the same breast, and the incidence of acute mastitis in this study (Table 4).

The correlation between 11 influencing factors and the incidence of acute mastitis was analyzed by one-way ANOVA. The variance of “primiparity age,” “mode of delivery,” and “frequency of nipple cleansing” was consistent with homogeneity of variance. For factor analysis of variance, there were significant differences in “primiparity age” and “frequency of nipple cleansing” between the two groups (*p* < 0.05). According to the level of *α* = 0.05, we can conclude that there were significant differences between the case group and the control group in the influence factors of primiparity age and frequency of nipple cleansing on the incidence of acute mastitis, and the correlations were statistically significant in this study.

### 3.4. Logistic Regression Subgroup Analysis for Nipple Infection, Improper Diet, and Emotional Stimulation

The study also statistically accounted for known lifestyle risk factors for acute mastitis such as nipple infection, improper diet, and stress by logistic regression subgroup analysis (Table 5).

The results of Forward Stepwise Regression for subgroups of nipple infection, improper diet, and emotional stimulation showed that milk pump damage (OR, 13.529; 95%CI: 3.094, 59.159) and infant bite (OR, 2.863; 95%CI: 1.460, 5.615), spicy food (OR: 5.420; 95%CI: 1.499, 19.598), *warm* fruit (OR: 5.420; 95%CI: 1.499, 19.598), *warm* meat and broth (OR: 3.042; 95%CI: 1.738, 5.323), and melancholy (OR: 3.043; 95%CI:1.675, 5.526) can be considered as risk factors for the occurrence of acute mastitis. We performed one-way ANOVA to analyze the correlation between “milk pump damage” (or “Lactagogue food”) and the incidence of acute mastitis, and the results showed that there were no significant differences in “milk pump damage” and “Lactagogue food” between the two groups (*p*=0.283 and *p*=0.165) according to the test level of *α* = 0.05. Therefore, we concluded that the correlation between “Milk pump damage” and the incidence of acute mastitis was not statistically significant in this study, as well as “Lactagogue food”.

### 3.5. Distribution of Constitution of TCM

A total of 24 (14.8%) participants in the case group were classified as BC. The frequency of biased constitution from high to low in the case group was QSC, QDC, Yin-Deficiency Constitution (YIDC), Yang-Deficiency Constitution (YADC), Phlegm-Dampness Constitution (PDC), Blood-Stasis Constitution (BSC), Dampness-Heat Constitution (DHC), and Inherited Special Constitution (ISC). A total of 70 (67.3%) participants in the control group were classified as BC. The frequency of biased constitution from high to low in the control group was QSC, YIDC, YADC, BSC, PDC, DHC, and QDC.

A total of 77 patients in the case group had acute mastitis within 8 weeks postpartum. The frequencies of the biased constitution from high to low of those specific patients were QDC, QSC, YIDC, YADC, PDC, DHC, BSC, and ISC. QDC and QSC accounted for more than 50%. A total of 30 patients in the case group have acute mastitis within 25–48 weeks postpartum. The frequencies of the biased constitution from high to low of those specific patients were QSC, QDC, PDC, YIDC, YADC, DHC, and BSC. ISC, QDC, and QSC accounted for more than 50%.

### 3.6. Logistic Regression Analyzing Constitution of TCM Affecting Incidence of Acute Mastitis

After introducing 9 constitutions of TCM by Forward Stepwise Regression, 2 potential risk factors, which were BC and QDC, were screened out. The OR value and its 95% CI of “BC” were 0.314 and (0.202, 0.487), respectively. Therefore, it can be considered as a protective factor for the occurrence of acute mastitis, while QDC (OR, 2.605; 95%CI: 1.393, 4.871) was a risk factor (Tables 6 and 7).

### 3.7. Cluster Analysis of Constitution of TCM

Cluster analysis of the constitution of TCM is shown in Figures 2 and 3. The 9 constitutions of TCM in the control group were divided into three categories. The first category was BC, the second category was QSC, and the rest 6 TCM constitution types were classified to the third category. The 9 constitutions of TCM in the case group were also divided into three categories. The first category was BC, the second category was QSC and QDC, and the rest 5 types were classified to the third category.

The 9 constitutions of TCM in the control group were divided into six categories. The first category was BC. The second category was QDC. DHC, PDC, BSC, and ISC belonged to the third category, while YADC, YIDC, and QSC were classified to the fourth, fifth, and sixth categories, respectively. The 9 constitutions of TCM in the case group were divided into six categories. The first category was BC. The second category was QDC and QSC. The third category was PDC and YIDC, while YADC and DHC were classified into the fourth and the fifth categories, respectively. BSC and ISC belonged to the sixth category.

The 9 constitutions of TCM in the control group were divided into five categories. The first category was BC while YIDC, YADC, and QSC were classified into the second, third, and fourth categories, respectively. BSC, ISC, DHC, PDC, and QDC belonged to the fifth category. The 9 constitutions of TCM in the case group were divided into five categories. The first category was BC. The second category was QSC and QDC, while YADC and DHC were classified into the third and fourth categories, respectively. The ISC, BSC, YIDC, and PDC were classified into the fifth category.

### 3.8. Changes of Symptoms in Biased Constitution of Traditional Chinese Medicine Postpartum

We added “whether the situation changed after delivery, including mitigation, no change, and aggravation” after each item of Self-Test Table” in the questionnaires for the case group, and postpartum problems were analyzed by changes in conversion score according to TCM type self-rating table of the constitution of TCM (ZYYXH/T157-2009) [18].

Some of the participants with BC (non-biased constitution type) had 1–3 symptoms related to one specific type of biased constitution aggravated; the frequency from high to low was BSC, QDC, YIDC, DHC, QSC, YADC, and ISC. Among patients with BC who had more than 4 symptoms related to one specific type of biased constitutions aggravated, only QSC accounted for 6% and the rest of other biased constitutional types accounted for less than 5%, respectively (Figure 4).

Meanwhile, some patients with BC had 1–3 symptoms related to one specific type of biased constitution relieved. The frequency from high to low was PDC, YIDC, YADC, QIDC, DHC, BSC, QSC, and ISC. Among patients with BC who had more than 4 symptoms related to one specific type of biased constitutions relieved, all biased constitutional types accounted for less than 5% each (Figure 5).

Among participants with biased constitution type who had 1–3 symptoms related to one specific type of biased constitutions aggravated, the frequency from high to low was QSC, QDC, PDC, BSC, YIDC, DHC, YADC, and ISC. Among those who had 4–6 symptoms related to one specific type of biased constitutions aggravated, the frequency from high to low was QSC, QDC, DHC, YIDC, PDC, YADC, BSC, and ISC. Few patients in the case group had more than 7 symptoms related to one specific type of biased constitutions aggravated, which only occurred in those who had QDC, YADC, QSC, and PDC and accounted for less than 5%.

Among participants tended to possess biased constitution type who had 1–3 symptoms related to one specific type of biased constitutions aggravated. The frequency from high to low was QDC, BSC, PDC, QSC, YIDC, YADC, DHC, and ISC. Among those who had more than 4 symptoms related to one specific type of biased constitutions aggravated, only YIDC accounted for 7% and the rest of other biased constitutional types accounted for less than 5% each.

Among patients with biased constitution type who had 1–3 symptoms related to one specific type of biased constitution relieved, the frequency from high to low was DHC, QDC, QSC, PDC, YIDC, YADC, BSC, and ISC. Among those who had 4–6 symptoms related to one specific type of biased constitution relieved, only QDC accounted for 6% and the rest of other biased constitutional types accounted for less than 5%, respectively.

Among patients who tended to possess biased constitution type who had 1–3 symptoms related to one specific type of biased constitution relieved, the frequency from high to low was DHC, YADC, PDC, QDC, YIDC, BSC, QSC, and ISC. Among those who had more than 4 symptoms related to one specific type of biased constitution relieved, only QSC accounted for 7% and the rest of the other biased constitutional types accounted for less than 5%, respectively.

## 4. Discussion

Our results showed that there was no significant difference in the prevalence of bilateral breasts. The incidence of primipara was significantly higher than that of second births. The incidence of acute mastitis was mostly within 8 weeks postpartum and most commonly within 4 weeks postpartum, accounting for about 25% of the total sample in the case group.

Frequent nipples cleansing is one of the protective factors of incidence of acute mastitis. The 95%CI of variance “regular nipples cleansing” in logistic regression analysis only ranged from 0.350 to 0.671 in this study, which suggested that a larger sample size was needed to confirm it. Our results were consistent with previous literature [9, 11], and both suggested that regular nipples cleansing was beneficial to reducing the probability of bacterial growth in the nipples.

Our results indicated that the most relevant risk factor for acute mastitis was nipple infection, and subgroup analysis further showed that milk pump damage was the most important risk factor during breastfeeding, followed by infant bite. Acute mastitis is an inflammation within the ducts of the breast as well as the connective tissue around them. Breastfeeding exposed the ducts of the breast, a relatively confined internal environment, to exoteric air. Damage caused by milk pump or sucking injury of infant bite may result in damage of papillary epidermal cells and loss of protective wounds, which made nipple and areola an ideal breeding ground for bacteria. According to our findings, the correlation between the usage of milk pumps and acute mastitis was not statistically significant. Whether milk pump affects acute mastitis is a controversial issue. Some scholars have found that it plays an important role in promoting milk secretion [19, 20]. A Spanish study has reported the use of breast pumps as a risk factor for mastitis [8]. Milk pump should be applied combined with the right way of breast massage and lactation instead of overuse. Therefore, lactating women should be guided by professional health care providers to know the correct way to use milk pumps properly. Dermatitis and rash in nipple-areola area, papillary bleb pricking or other trauma, and babies falling asleep with nipple bitten may directly or indirectly cause local nipple infection, which was inconsistent with some studies [8, 21, 22]. However, the correlation between these three factors and the incidence of disease was not statistically significant in our study due to the limited sample size of each item.

Primiparous and later primiparity age might contribute to the incidence of acute mastitis. The average primiparity age in the case group was 30 years, and that in the control group was 28 years, which was slightly earlier than those in the case group. Leila et al. [7] have found that primiparity age over 30 years old and parturient woman over 30 years old are the risk factors of mastitis or even breast abscess. Xia and Yang [23] believed that primipara's milk contained more exfoliated epithelial cells, which can easily lead to blockage of the duct and aggravate milk deposition. Through questionnaires, Cheng et al. [24] concluded that lacking lactation experience and good breastfeeding habits and failing to grasp the method of breastfeeding correctly were common problems among Chinese young mothers.

The delivery mode was a related risk factor that contributed to the incidence of acute mastitis; whether the cesarean section was a protective or risk factor for acute mastitis remained a question and still debated in the literature [5, 25]. In our study, cesarean section was a protective factor for the incidence of the disease compared with vaginal delivery. Domestic scholar Chen's study had the opposite conclusion [26]. Considering the 95% CI of OR value was only 0.322–0.910 and there was no significant difference between the case group and the control group based on one-way ANOVA analysis, the conclusion needed to be verified by further study with an expanded sample size.

Interestingly, we found that acute mastitis often occurred within 8 weeks postpartum; another peak was 6–7 months postpartum, accounting for about 18% in the case group. The reason for the peak is that many young mothers return to work 5–6 months postpartum. The adjustment was hard during the first month after going back to the workforce; some suffered from this disease during the process of delectation. Stress, physical fatigue, and negative emotions like melancholy can cause the decline of sIgA level, which leads to the decrease of body resistance to bacteria and susceptibility to infectious diseases, such as mastitis by influencing the immune system [26, 27].

The establishment of the first maternal-infant connection as soon as possible after delivery is conducive to prevent acute mastitis, [8] which is accorded with our results. The later the time of colostrum secretion, the greater the risk of acute mastitis; the incidence of postpartum colostrum after 72 h was 1.7 times higher than that of postpartum colostrum within 24 h.

A total of 29.6% of the subjects in the case group were or were prone to be BC, and the frequency distribution of biased constitutions (subjects classified as “Yes” or “Prone to be”) from high to low was QSC, QDC, YIDC, YADC, PDC, DHC, BSC, and ISC. The proportion of QSC and QDC was up to 59.5%. A total of 88.5% of the participants in the control group were or were prone to be BC. The most common biased constitution types with the highest frequency of distribution were QSC, YIDC, and YADC, accounting for 17.3%, 10.5%, and 9.6%, respectively. It can be inferred that more participants were or were prone to be BC in the control group than in the case group and more subjects with biased constitution type in the case group than the control group.

QSC, YIDC, and YADC were of the highest frequency of distribution in both the case group and the control group. Cluster analysis showed that dysfunction of Qi, mainly manifested as Qi-Deficiency and Qi-Stagnation, was more common in the case group than in the control group. In accordance with the results of regression analysis, the protective factor of acute mastitis was BC, while the risk factor was QDC. According to TCM Theory, Qi-Deficiency and Qi-Stagnation depended on each other and mutually transformed into each other. It was in step with previous domestic research which highlighted the importance of Qi and blood dysfunction [28–30]. However, our research made the further deduction that QDC was a risk factor of acute mastitis. Although the correlation between QSC and the incidence of the disease had not been statistically significant in this study, QSC might be a potential risk factor for acute mastitis.

In order to explore the postpartum change of biased constitution type among breastfeeding mothers, we analyzed alleviation and aggravation of their biased constitution type-related symptoms before and after delivery. Whether the subjects were classified as the constitution type or not, more than one-third of the total subjects had no significant change of biased constitution type-related symptoms after delivering babies. The participants with QSC, QDC, PDC, and BSC were more likely to have 1–3 symptoms aggravated while four or more symptoms aggravated accounted for less than 20%. The aggravation of the rest biased constitution type was not obvious. As for their alleviation of various biased constitution type-related symptoms, DHC was most common in those with 1–3 related symptoms alleviated. PDC-related symptoms had 4 or more items alleviated but accounted for less than 10% of total cases, which did not have statistical significance.

It seemed that most patients did not significantly change with symptoms of various constitutions of TCM after delivery. Among the patients with some changes, the symptoms of QSC, QDC, PDC, and BSC were aggravated. Qi and blood were two important basic elements of vital energy; postpartum women consumed a lot of vital energy, such as Qi, Yin, and blood after delivering, breastfeeding, and taking care of babies. Pressure from work and family, inappropriate diet, and inadequate sleep are influencing factors that lead to organ dysfunction and poor Qi-blood circulation such as Qi-Stagnation, Qi-Deficiency, and Blood-Stasis. Poor Qi and blood circulation turbulence spleen and liver's as well as mid-Jiao's function results in accumulation of phlegm, dampness, and unfavorable heat. Therefore, lactating women are prone to have Qi and blood dysfunction as well as relevant symptoms of QSC, QDC, PDC, and BSC. Those symptoms may aggravate after delivery, thereby increasing the onset of acute mastitis.

Participants who were with DHC and PDC were more likely to have symptoms relieved. Some scholars even believed that DHC and PDC were risk factors for acute mastitis [28–31]. It may be related to both exogenous dampness (such as lower air humidity after delivery) and internal dampness (such as consuming too much fatty meat and broth or spicy food), but the correlation among them was inconclusive due to limited sample size. People with DHC or PDC were suggested to avoid consuming too much spicy food and fatty meat or broth that obstructed mammary glands and its related meridians in the previous literature [28–31].

When analyzing the relationship between acute mastitis and the constitution of TCM and the potential risk factors of acute mastitis in Chinese breastfeeding mothers, we found that the first peak occurred in the short term after delivery, due to the deficiency of Qi and blood, the two important basic elements of vital energy. Breastfeeding mothers with QDC were susceptible to acute mastitis, physical fatigue, and more nutrition demanding and consuming resulting in immune and neuroendocrine changes and vulnerability to bacterial infection [27, 31]. QDC was a risk factor of acute mastitis of this period while the second peak occurred when most lactating women returned to work. Facing the double pressures of family and work, those women who choose to continue lactating may experience emotional changes such as tension, anxiety, and depression. According to theories of TCM, emotional changes may interfere with the function of organs and meridians as well as mammary glands, leading to poor Qi and blood circulation and accumulation of milk. Therefore, QSC and BSC were more likely to be the risk factors for mastitis of the second peak. It was consistent with the conclusion that negative emotion resulted in a decline in the body's resistance to bacteria [26, 31].

This finding might be a reference for clinical practice, where the prognosis of patients with acute mastitis can be identified by TCM constitution type and its relevant symptoms. For example, people with QDC and BC have quite different clinical manifestations. People with Qi-Deficiency symptoms have the following characteristics: (i) general manifestations: lack of vitality, fatigue, shortness of breath, and self-sweating; (ii) physical characteristics: soft and loose muscles; (iii) common manifestations: with a weak voice and low spirits, light red tongue, tooth marks on the edge of the tongue, and weak pulse; (iv) psychological characteristics: introverted and not willing to take risks; (v) incidence tendency: easy to suffer from cold, visceral ptosis, and other diseases and difficult to recover after illness; (vi) adaptability to the external environment: intolerant to wind, cold, heat, and dampness. However, people with Balanced Constitution might have opposite symptoms: (i) energetic, not easy to fatigue, and tolerance to cold and heat; (ii) good appetite and robust body; (iii) dense and shiny hair, vivid eyes, bright nose and ruddy lips, light red tongue, thin and white moss, and mild pulse; (iv) easygoing and cheerful characteristics; (v) not easy to get sick and easy recovery after illness; (vi) strong adaptability to the natural environment and social environment [29].

## 5. Conclusion

1. The protective factors of acute mastitis were regular nipple cleansing and cesarean section. The risk factor was nipple infection. For patients with all constitutions of TCM, regular nipple cleansing and breast vacuuming can avoid nipple infection, and a healthy lifestyle and positive mental state can prevent acute mastitis attack
2. Among all the constitutions of TCM, BC was a protective factor, while QDC was a risk factor
3. The breastfeeding mothers with acute mastitis were more likely to have deficiency symptoms and constitution types within 6–8 postpartum, ”tonifying Qi and blood” should be stressed. While the second peak occurred soon after they returned to work, negative emotions and pressure may lead more patients to have QSC and BSC. Avoiding overthinking and controlling negative feelings were good ways to soothe Qi-Stagnation and promote Qi-blood circulation, thus reducing the occurrence and deterioration of the disease

## Figures and Tables

**Figure 1:** Distribution of the onset time of acute mastitis.

**Figure 2:** Icicle plots of constitution types in traditional Chinese medicine in the case and the control group. The horizontal axis represents nine types of TCM constitution types clustered, while the vertical axis indicates that these nine types of constitution are clustered into several categories, which demonstrated the classification results of TCM constitution types when clustered into different categories.

**Figure 3:** Dendrogram of constitution of TCM in the case and the control group. The horizontal axis represents the relative distances of various categories after clustering, which is a general change of the distances between categories; the vertical axis is the object of clustering.

**Figure 4:** Distribution of biased physical symptoms in postpartum whose symptoms were aggravated.

**Figure 5:** Distribution of biased physical symptoms in postpartum whose symptoms were relieved.

**Table 1:** Judging criteria of the constitution of TCM.

Constitution of TCM	Score	Results
Balanced constitution	Conversion score ≥60 points	Yes
	All biased constitution type's conversion score <30 points	
	Conversion score ≥60 points	Prone to be
	All biased constitution type's conversion score <40 points	
	All the above-mentioned conditions not satisfied	No

Biased constitution type	Conversion score≥40 points	Yes
	Conversion score 30–39 points	Prone to be
	Conversion score＜30 points	No

**Table 2:** Baseline demographic characteristics between the two groups.

Variables		Case group	Control group	*P* value
		*N* = 184 (%)	*N* = 201 (%)	
Educational background	High school or below	5 (2.7%)	13 (6.5%)	0.194
	University or college graduates	142 (77.2%)	153 (76.1%)	
	Master or doctor degree	37 (20.1%)	35 (17.4%)	

Previous history of benign breast diseases	Yes, with prenatal history of breast surgery	8 (4.3%)	6 (3.0%)	0.332
	Yes and without a prenatal history of breast surgery	28 (15.3%)	22 (10.9%)	
	No	148 (80.4%)	173 (86.1%)	

Family history of acute mastitis	Yes	4 (2.2%)	0 (0%)	0.051
	No	180 (97.8%)	201 (100%)	

Previous history of breast tumors	Benign	4 (1.6%)	3 (1.5%)	0.587
	Malignant	4 (1.6%)	2 (1%)	

**Table 3:** Distribution of maternity or lactation-related factors between the two groups.

Variables		Case group	Control group	*P* value
		*N* = 184 (%)	*N* = 201 (%)	
Parity	Primipara	157 (85.3%)	188 (93.5%)	0.008
	Multipara	27 (14.7)	13 (6.5%)	

Primiparity age	18–28 years old	62 (33.7%)	113 (56.2%)	<0.001^*∗∗*^
	29–35 years old	110 (59.8%)	83 (41.3%)	
	36–45 years old	12 (6.5%)	5 (2.5%)	

Mode of delivery	Vaginal delivery	102 (55.4%)	110 (54.7%)	0.845
	Cesarean section	80 (43.5%)	90 (44.8%)	
	Delivery with forceps	2 (1.1%)	1 (0.5%)	

Fetal status	Fetal full-term	149 (81.0%)	193 (96.0%)	<0.001^*∗∗*^
	Preterm birth	16 (8.7%)	5 (2.5%)	
	Fetal overdue birth	19 (10.3%)	3 (1.5%)	

Postpartum colostrum	≤24 hours	75 (40.8%)	126 (62.7%)	<0.001^*∗∗*^
	25–48 hours	44 (23.9%)	57(28.3%)	
	49–72 hours	46 (25%)	13 (6.5%)	
	≥72 hours	19 (10.3%)	5 (2.5%)	

First lactation time after delivery	≤24 hours	79 (42.9%)	111(55.2%)	<0.001^*∗∗*^
	25–48 hours	40 (21.7%)	62 (30.8%)	
	49–72 hours	35 (19.0%)	19 (9.5%)	
	≥72 hours	30 (16.3%)	9 (4.5%)	

Times of breastfeeding each day	≤2 times	7 (3.8%)	1 (0.5%)	<0.001^*∗∗*^
	3–6 times	88 (47.8%)	143 (71.1%)	
	≥7 times	89 (48.4%)	57 (28.4%)	

Time of consecutive feeds with same breast	≤10 minutes	17 (9.2%)	8 (4.0%)	<0.001^*∗∗*^
	10–15 minutes	80 (43.5%)	61 (30.3%)	
	16–30 minutes	70 (38.0%)	128 (63.7%)	
	≥30 minutes	17 (9.2%)	4 (2.0%)	

Milk yield	Insufficient	54 (29.4%)	45 (22.4%)	0.285
	Adequate or redundant	111 (60.3%)	135 (67.2%)	
	Surplus	19 (10.3%)	21 (10.4%)	

Milk pump damage	Yes	152 (82.6%)	174 (86.6%)	0.281
	No	32 (17.4%)	27 (13.4%)	

Lactagogue food	Yes	74 (40.2%)	95 (47.3%)	0.164
	No	110 (59.8%)	106 (52.7%)	

Crater nipple	Yes	34 (18.5%)	43 (21.4%)	0.475
	No	150 (81.5%)	158 (78.6%)	

Times of nipple cleansing each day	≤1 times	79 (43.0%)	35 (17.4%)	<0.001^*∗∗*^
	2–3 times	58 (31.5%)	60 (29.9%)	
	≥4 times	47 (25.5%)	106 (52.7%)	

^∗∗^ *P* < 0.001 between the groups.

**Table 4:** Multivariable Logistic Regression analysis of risk factors for acute mastitis.

Variables	*B*	Wald *X*^2^	*P*	OR	95% CI for EXP (B)	
					Lower	Upper
Primiparity age	0.126	10.306	0.001	1.135	1.050	1.226
Mode of delivery	−0.613	5.365	0.021	0.541	0.322	0.910
Postpartum colostrum	0.555	12.680	<0.001^*∗∗*^	1.742	1.283	2.364
Times of breastfeeding each day	0.389	4.653	0.031	1.475	1.036	2.100
Frequency of nipple cleansing	−0.725	19.059	<0.001^*∗∗*^	0.484	0.350	0.671
Nipple infection	1.964	37.573	<0.001^*∗∗*^	7.128	3.804	13.357
Improper diet	1.273	17.500	<0.001^*∗∗*^	3.573	1.967	6.488
Emotional stimulation	0.658	4.606	0.032	1.930	1.059	3.519
Parity	1.620	13.177	<0.001^*∗∗*^	5.053	2.107	12.118
Constants	−4.735	12.903	<0.001^*∗∗*^	0.009	—	—

^∗∗^ *P* < 0.001 between the groups.

**Table 5:** Logistic regression subgroup analysis for nipple infection, improper diet, and emotional stimulation.

Variances		b	Wald *X*^2^	*P*	OR	95% CI for EXP (B)	
						Lower	Upper
Nipple infection	Infant bite	1.052	9.375	0.002	2.863	1.460	5.615
	Milk pump damage	2.605	11.973	0.001	13.529	3.094	59.159

Improper diet	Spicy food	1.690	6.642	0.010	5.420	1.499	19.598
	*warm* ^*∗*^fruit	1.690	6.642	0.010	5.420	1.499	19.598
	*warm* ^*∗*^meat and broth	1.112	15.181	<0.001^*∗∗*^	3.042	1.738	5.323

Emotional stimulation	Melancholy	1.113	13.355	<0.001^*∗∗*^	3.043	1.675	5.526

^*∗*^ *Warm* food was defined as food having “warm, bright, or outward” attributes, such as spicy food, fatty meat, or broth and fruits like orange, dates, and bayberries, according to traditional Chinese medicine (TCM). ^∗∗^*P* < 0.001 between the groups.

**Table 6:** Binary logistic regression analysis of risk factors for acute mastitis in the constitution of TCM.

Variances	*B*	Wald *X*^2^	*P* value	*OR*	95% CI for EXP (B)	
					Lower	Upper
BC	−1.021	9.558	0.002	0.360	0.189	0.688
QDC	0.931	7.519	0.006	2.536	1.304	4.933
YADC	0.061	0.038	0.845	1.063	0.575	1.966
YIDC	−0.028	0.007	0.935	0.973	0.500	1.893
PDC	0.132	0.116	0.734	1.141	0.534	2.440
DHC	0.562	1.481	0.224	1.755	0.709	4.341
BSC	0.027	0.004	0.949	1.027	0.451	2.341
QSC	−0.056	0.031	0.861	0.945	0.505	1.769
ISC	0.295	0.222	0.638	1.343	0.394	4.575
Constants	0.913	2.364	0.124	2.491	—	—

**Table 7:** Multivariable logistic regression analysis of risk factors for acute mastitis in the constitution of TCM.

Variances	*B*	Wald *X*^2^	*P* value	*OR*	95% CI for EXP (B)	
					Lower	Upper
BC	−1.158	26.701	<0.001^*∗∗*^	0.314	0.202	0.487
QDC	0.958	8.992	0.003	2.605	1.393	4.871
Constants	1.190	11.354	0.001	3.286	—	—

^∗∗^ *P* < 0.001 between the groups.

## Data Availability

Nondigital data supporting this study are stored by the corresponding author at the Shanghai University of Traditional Chinese Medicine. Details of how to access these data are provided in the documentation available at Shanghai University of Traditional Chinese Medicine.

## Abbreviation

TCM: Traditional Chinese medicine
QSC: Qi-Stagnation Constitution
BC: Balanced Constitution
PDC: Phlegm-Dampness Constitution
YADC: Yang-Deficiency Constitution
DHC: Dampness-Heat Constitution
YIDC: Yin-Deficiency Constitution
BSC: Blood-Stasis Constitution
QDC: Qi-Deficiency Constitution
ISC: Inherited special constitution
OR: Odds ratio
CI: Confidence interval.
